# Efficient COVID-19 CT Scan Image Segmentation by Automatic Clustering Algorithm

**DOI:** 10.1155/2022/9009406

**Published:** 2022-03-30

**Authors:** Basu Dev Shivahare, S. K. Gupta

**Affiliations:** ^1^Department of Computer Science and Engineering, Dr. A.P.J Abdul Kalam Technical University, Lucknow, Uttar Pradesh, India; ^2^Department of Computer Science and Engineering, B.I.E.T., Jhansi, Uttar Pradesh, India

## Abstract

This article addresses automated segmentation and classification of COVID-19 and normal chest CT scan images. Segmentation is the preprocessing step for classification, and 12 DWT-PCA-based texture features extracted from the segmented image are utilized as input for the random forest machine-learning algorithm to classify COVID-19/non-COVID-19 disease. Diagnosing COVID-19 disease through an RT-PCR test is a time-consuming process. Sometimes, the RT-PCR test result is not accurate; that is, it has a false negative, which can cause a threat to the person's life due to delay in starting the specified treatment. At this moment, there is an urgent need to develop a reliable automatic COVID-19 detection tool that can detect COVID-19 disease from chest CT scan images within a shorter period and can help doctors to start COVID-19 treatment at the earliest. In this article, a variant of the whale optimization algorithm named improved whale optimization algorithm (IWOA) is introduced. The efficiency of the IWOA is tested for unimodal (F1–F7), multimodal (F8–F13), and fixed-dimension multimodal (F14–F23) benchmark functions and is compared with the whale optimization algorithm (WOA), salp swarm optimization (SSA), and sine cosine algorithm (SCA). The experiment is carried out in 30 trials and population size, and iterations are set as 30 and 100 under each trial. IWOA achieves faster convergence than WOA, SSA, and SCA and enhances the exploitation and exploration phases of WOA, avoiding local entrapment. IWOA, WOA, SSA, and SCA utilized Otsu's maximum between-class variance criteria as fitness function to compute optimal threshold values for multilevel medical CT scan image segmentation. Evaluation measures such as accuracy, specificity, precision, recall, *G*mean, F_measure, SSIM, and 12 DWT-PCA-based texture features are computed. The experiment showed that the IWOA is efficient and achieved better segmentation evaluation measures and better segmentation mask in comparison with other methods. DWT-PCA-based texture features extracted from each of the 160 IWOA-, WOA-, SSA-, and SCA-based segmented images are fed into random forest for training, and random forest is tested with DWT-PCA-based texture features extracted from each of the 40 IWOA-, WOA-, SSA-, and SCA-based segmented images. Random forest has reported a promising classification accuracy of 97.49% for the DWT-PCA-based texture features, which are extracted from IWOA-based segmented images.

## 1. Introduction

Image segmentation is the preprocessing step for analyzing a medical image and is utilized in classification applications. Important features such as texture and shape-based features are extracted from the segmented image. COVID-19 is highly contagious and spreads through contact and respiratory illness [1, 2]. It is a challenging task to determine COVID-19 disease in humans accurately through RT-PCR [3, 4] and rapid antigen kit. People who are affected by coronavirus may feel symptoms such as trouble in breathing, chest pain, belly pain, and pressure in the chest. Diagnosing COVID-19 disease via RT-PCR is a time-consuming process, and when coronavirus cases were at the peak, the RT-PCR test results were available 48 hours after the sample collection. Since treatment can only be started after obtaining the result, people have to wait till the disease reach studies its worst level, significantly increasing the chances of death. Sometimes, the RT-PCR test is not accurate; that is, has a false result, then it may be a threat to a person's life due to the late start of specified treatment. As per the above scenario, there is an urgent need to develop a reliable automatic COVID-19 detection tool that detects COVID-19 disease from chest CT scan images within a shorter time and may help doctors to start COVID-19 treatment at the earliest. Chiranji Lal et al. [5] discussed various medical imaging modalities and surveyed various segmentation techniques. Manual medical image segmentation by a medicinal professional is a time-consuming process, and the diagnosis might be erroneous. Sonam Aggarwal et al. [6] have made comparative analysis among various pretrained DL models for detection and classification of COVID-19 from normal and pneumonia images. Shiv Naresh et al. [7] applied the region-based active contour method and convex hull approach to segment and detect brain tumours from the BRATS 2015 dataset. The average sensitivity, PPV, and DSC were 92% for a complete brain tumour, 83% for an enhanced brain tumour, and 81% for brain tumour core. Adnan Saood et al. [8] utilized U-net and SegNet to segment COVID-19 lung CT scan images. SegNet achieved 95% mean accuracy in classifying infected/noninfected tissues. Arjun Sarkar et al. [9] used Vision Pro and Cognex DL software classified chest X-ray from the COVIDx dataset. Vision Pro achieved a 95.3% F-score on a segmented image and 94% on the entire image as ROI and performed better than COVID-Net. Nilesh Bhaskarrao Bahadure et al. [10] applied Berkeley wavelet transformation for brain tumour segmentation, and extracted features from the segmented images were utilized by SVM to classify into normal/abnormal tissue. Shaoqiong Huang et al. [11] applied DL-based attention Gabor network (Agnet) for lung segmentation, which achieved better segmentation accuracy in FMLCD and LiTS datasets than FCN, U-Net, U-Net++, and Attention U-Net. Saumya Ranjan et al. [12] utilized pretrained DL models to detect COVID-19/normal from chest X-ray images. The proposed method with various pretrained DL models accuracy varies between 92.50% and 98.33%. The proposed method with Res-net 34 achieved 98.33% accuracy. Armando Ugo Cavallo et al. [13] extracted 308 texture features per ROI from chest X-ray and analyzed pneumonia infection in COVID-19 patients using machine-learning models. Metaheuristic algorithms [14] are becoming more popular because they do not require gradient information, have ability to avoid entrapment into local optima, and are utilized to solve complex optimization problems efficiently. Mohamed Abd El Aziz et al. [15] presented Moth Flame optimization and WOA separately using the Otsu method for multilevel thresholding image segmentation. The best fitness result, time complexity, and segmentation quality metrics of PSNR, SSIM, and ANOVA tests were computed for WOA, MFO, and other swarm-based algorithms. WOA and MFO performed better than other algorithms. A.A.Ewees et al. [16] proposed the whale optimization algorithm (WOAMOP) with Otsu's and Kapur's entropy utilized as the fitness function to determine the optimal set of thresholds. The proposed method has been compared with WOA, FA, Social Spider Optimization (SSO), and FASSO. The average fitness result, CPU processing time, multilevel threshold values, SSIM, and PSNR were evaluated over 30 runs and 100 iterations for the proposed method along with other algorithms. WOAMOP achieved better segmentation quality metrics PSNR and SSIM for threshold number *k* = 2,3,4, and 5. Seyedali Mirjalili et al. [17] proposed salp swarm algorithm (SSA) and multiobjective problems are solved by multiobjective salp swarm algorithm. The SSA first explores the search space and then performs the exploit phase. In the SSA, the position of follower salps is updated to achieve the global position. The efficiency of the SSA is tested on F1–F19 benchmark functions for 30 trials, population size is set as 30 and 500 iterations in each run, and the statistical results such as standard deviation and mean are compared with PSO, GSA, BAT, flower pollination algorithm (FPA), SMS, firefly algorithm (FA), and genetic algorithm (GA). The SSA is able to explore the most promising area of problems and obtains better mean standard deviation values and outperforms in majority of unimodal, multimodal, and composite test functions. Seyedali Mirjalili [18] proposed a sine cosine algorithm (SCA) to solve optimization problems. The efficiency of the SCA is tested on F1–F19 benchmark functions for 30 trials, the population size is set as 30 and 500 iterations in each run, and the statistical results such as standard deviation and mean are compared with PSO, GA, BAT, and Flower Pollination Algorithm (FPA). The SCA establishes a balance between exploration and exploitation to find global optima and achieves fast convergence behavior than the other algorithms. BD Shivahare and S.K.Gupta [19] applied a randomized spiral phase-based whale optimization algorithm and evaluated multilevel optimal threshold and segmentation metrics such as PSNR, SSIM, MSE, and average difference. Kapil Kumar Gupta et al. [20] proposed hybrid K-means clustering and fuzzy C means algorithm for brain tumour segmentation and classification of benign/malignant brain tumours. V.Viswa Priya and Shobarani [21] proposed a contextual clustering algorithm to perform brain tumour segmentation. A. Renugambal and K. Selva Bhuvaneswari [22] applied hybrid water cycle moth flame optimization to obtain optimal thresholds for brain MR image segmentation. Otsu's maximum between-class variance criteria are utilized as the objective function. WCMFO has achieved a fast convergence rate to compute optimal thresholds and has improved quantitative metrics such as PSNR, CPU time, and std. deviation. Mohammad Hashem Ryalat et al. [23] applied PSO, DPSO, and FODPSO algorithms on three brain tumour MR images, performed segmentation and volume reconstruction, and identified tumours that affected the head and neck. FODPSO has performed better than others in terms of speed, accuracy, and stability. Dilbag Singh et al. [24] proposed a MADE-based deep convolution neural network model to diagnose COVID-19 disease from chest X-rays. Multiobjective adaptive differential evolution (MADE) is used to overcome hyperparameters tuning issues of the deep convolution neural network. The accuracy of the proposed model ranges between 93% and 97%. El abbadi, Nidhal & Faisal, Zahraa [25] proposed a method to segment brain tumour and classification. The authors used 3-level DWT to extract features from tumour-detected region and utilized the PCA to reduce the dimensions of features. Twenty brain MRI images and 45 brain MRI images were used to train and test ANN, respectively. Thirteen statistical and texture features were used as input to ANN for classification. Abdalla Mostafa et al. [26] applied the whale optimization algorithm to compute various clusters and utilized statistical images for liver image segmentation. Maximum, minimum, and average quantitative metrics such as accuracy, SSIM, precision, and si are evaluated. Mohamed Abd Elaziz et al. [27] proposed density peak clustering with general extreme values (DPCGEVs) on 12 COVID-19 CT scan images to compute optimal thresholds. The proposed algorithm was compared with K-means and DPC and has performed better in terms of entropy, SSIM, and PSNR. Image Segmentation is a preprocessing step. The classification task is performed by a machine-learning model based on extracted features of the segmented image.

To analyze and diagnose disease from medical imaging through manual segmentation is a time-consuming process. In the field of medical science, a huge number of medical images are generated by computer-aided devices every day; therefore, it is very difficult to analyze and diagnose these medical images efficiently with manual segmentation method. Deep learning (DL) approaches are widely used in the medical image segmentation field. DL models [27] require vast training using a huge number of images and may not report good accuracy due to a limited number of images, and unsupervised machine-learning approaches such as clustering algorithms do not require training for images and are suitable to compute thresholds for multilevel image segmentation [17–19]. DL models suffer from hyperparameters tuning setting and overfitting issues. To overcome these issues, Kaur et al. [28] proposed a metaheuristic-based DL model to diagnose COVID-19 disease.

In this article, the authors propose a variant of the whale optimization algorithm named improved whale optimization algorithm (IWOA) utilizing the Otsu thresholding method as the fitness function to compute optimal thresholds for multilevel image segmentation. The efficiency of the proposed method, IWOA, has been compared with other nature-inspired metaheuristic algorithms such as whale optimization algorithm, salp swarm algorithm, and sine cosine algorithm on 23 benchmark functions as described in Section 4.2. The IWOA achieves faster convergence than others, enhances the exploitation and exploration phase of WOA, and avoids local entrapment. Each of metaheuristic algorithms such as IWOA, WOA, SSA, and SCA utilized Otsu's maximum between-class variance criteria as the objective function to compute optimal threshold values at threshold number *k* = 3 on 200 COVID-19 and normal chest CT scan images for multilevel image segmentation. Two-level DWT with the Haar wavelet filter is used to extract the features from the segmented image, and then, the PCA is used to reduce dimensions of features. Twelve DWT-PCA-based texture features are extracted from the segmented image and used as input into the random forest machine-learning algorithm for classification. The experiments have been conducted on 200 COVID-19 and normal chest CT scan images for image segmentation at threshold number *k* = 3, described in Section 4.3. Performance of the proposed image segmentation method and other algorithms has been analyzed using 21 parameters such as fitness score, optimal threshold values, and segmentation quality metrics such as structural similarity index (SSIM), accuracy, sensitivity, specificity, precision, F_measure, *G*mean, and 12 DWT-PCA-based texture features (Algorithm 1).

## 2. Materials and Methods

### 2.1. Problem Formulation

The aim of multilevel thresholding is to find best *k* threshold values, which are computed by Otsu's maximum between-class variance criteria. The Otsu method is used as fitness function and popular image thresholding method to determine multiple threshold values. Therefore, for *t*_*k*_, *k* = 1, 2, 3,…, *k* {*t*_1_, *t*_2_, *t*_3_,…, *t*_*k*_} thresholds, the image is segmented into *k* + 1 classes or levels. The range of each class is described as follows:

  Class1 = {*I* (*x*, *y*) *ε G* | 0 ≤ *G* (*x*, *y*) ≤ *t*_1_}
  Class2 = {*I* (*x*, *y*) *ε G* |*t*_1_ + 1 ≤ *G* (*x*, *y*) ≤ *t*_2_}
  ..…
  Class_*k*+1_ = {*I* (*x*, *y*) *ε G* | *t*_k_ + 1 ≤ *G* (*x*, *y*) ≤ *L* − 1}

Here, *I* (*x*, *y*) represents the intensity of pixel (*x*, *y*) of gray-level image *G* and *L* is gray levels *L ε* [0,255].

Best threshold values are computed by maximizing the following equation:

(1) $$\begin{array}{c} t_{1}^{*},t_{2}^{*},\ldots ,t_{T}^{*}=\text{maximize}\left\{t_{1},\;t_{2}\;,\ldots ,\;t_{T}\right\}\text{Fitness}\left(t_{1},\;t_{2},\ldots ,\;t_{T}\right)\text{,} \end{array}$$

where Fitness (*t*_1_,  *t*_2 _,…,  *t*_*T*_) is formulated as the following equation:

(2) $$\begin{array}{c} \text{ Fitness}\left(t_{1},\;t_{2\;},\ldots ,\;t_{T}\right)=\sum_{i=t_{1}}^{t_{T}}w_{i\;}\left({µ}_{i\;}-\;{µ}_{T}\right){\;}^{2}, \end{array}$$

where *w*_*i* _ and  *µ*_*i* _ represent the weight and mean of *i*th class, respectively, and  *µ*_*T*_ represents the total mean of the class. The weight of the *i*th class is given as follows:

(3) $$\begin{array}{c} w_{i\;}=\;\sum_{j=t_{i}}^{t_{i+1\;}-1}p_{j}. \end{array}$$

Here, *p*_*j*_  represents the probability of the *j*th class and defined as follows:

(4) $$\begin{array}{c} p_{j}=\frac{h\left(j\right)}{H}. \end{array}$$

Here, *h* (*j*) is the frequency of *j* gray level and *H* represents the total number of pixels.

The class means *µ*_*i*_ and *µ*_*T*_  are represented in the following equations, respectively:

(5) $$\begin{array}{c} {µ}_{i}\;=\;\sum_{j=t_{i}}^{t_{i+1\;}-1}i\;\frac{p_{j}}{w_{j}}, \end{array}$$

(6) $$\begin{array}{c} {µ}_{T}=\sum_{j=0}^{L-1}jp_{j}. \end{array}$$

The following conditions must be satisfied:

(7) $$\begin{array}{c} \overset{k+1}{\underset{i=1}{\sum }}w_{i\;}{µ}_{i\;}=\;{µ}_{T},\\ \overset{k+1}{\underset{i=1}{\sum }}w_{i\;}=\;1. \end{array}$$

### 2.2. Whale Optimization Algorithm

Mirjalili et al. [14] introduced the whale optimization algorithm (WOA), which is widely used to solve global optimization problem by emulating the humpback behavior. The WOA is gradient-free, avoids entrapment into local optima, and has ability to obtain optimal solution. Generally, these whales first encircle the target prey by forming bubbles of circular path or a path shaped like “9.” The WOA establishes the balance between exploration and exploitation phases. The exploration and exploitation phases performed by the WOA is described in Sections 2.2.1 and 2.2.2, respectively.

#### 2.2.1. Exploration Phase

In the exploration phase, whale is randomly selected from search space to obtain towards global or best position to obtain the close location of target prey. The position of whale is updated using the random position of whale $\overset{⟶}{X}$_rand_ for | $\overset{⟶}{A|}$ ≥ 1. The updated position of whale under the exploration phase is presented in the following equation:

(8) $$\begin{array}{c} \overset{⟶}{D1}=\;\left|\overset{⟶}{C}\text{.}{\overset{⟶}{X}}_{\text{rand}}-\overset{⟶}{X\left(t\right)}\right|,\\ \;\overset{⟶}{P}\left(\text{i }+\;1\right)={\overset{⟶}{X}}_{\text{rand}}-\overset{⟶}{A}\text{.}\overset{⟶}{D1}, \end{array}$$

where $\overset{⟶}{D1}\;$ is distance between current search agent $\;\overset{⟶}{X\left(t\right)}\;$ and randomly selected whale or search agent $\;\left({\overset{⟶}{X}}_{\text{rand}}\right)$ from search space.

#### 2.2.2. Exploitation Phase

In the WOA, the exploitation phase is performed by bubble net foraging behavior. Bubble creation behavior by humpback whale is done in two phases.

*(a) Shrinking Encircling Prey*. In this phase, the value of *a* is shrinking linearly from 2 to 0 over the successive iterations (*t*) and vector $\overset{⟶}{A}$ has a random value between [−1, 1] over the course of iterations. The encircling phase is expressed using the following equation:

(9) $$\begin{array}{c} \overset{⟶}{P}\left(i\;+\;1\right)={\overset{⟶}{X}}_{b}\left(i\right)-\overset{⟶}{A}.\overset{⟶}{D}, \end{array}$$

where $\overset{⟶}{P}$ (*i* + 1) represents the updated position of the search agent in *n* dimension at iteration *t* and ${\overset{⟶}{X}}_{b}$ is the positions of best search agent. Coefficient vector $\overset{⟶}{A}$ is mathematically defined in the following equation:

(10) $$\begin{array}{c} A=2\overset{⟶}{a}\cdot r-\overset{⟶}{a}. \end{array}$$

*D* denotes distance from the best agent, which is defined as follows:

(11) $$\begin{array}{c} D=\left|\overset{⟶}{C}.{\overset{⟶}{\;X}}_{b}\left(t\right)∼\overset{⟶}{X}\left(t\right)\right|. \end{array}$$

Here, $\overset{⟶}{X}\left(t\right)$ represents the positions of the search agent in search space at iteration *t*. Adjustment factor $\overset{⟶}{C}$ helps the search agents to exploit the local areas in search space and is defined as

(12) $$\begin{array}{c} \overset{⟶}{C}=2\cdot \text{r.} \end{array}$$

Here, *r* is a randomly generated number *r ε* (0, 1) and $\overset{⟶}{a}$ represents the vector.

*(b) Spiral Updating Position*. The updated position of search agents or whales under the spiral formation phase is mathematically expressed as

(13) $$\begin{array}{c} \overset{⟶}{P}\left(i\;+\;1\right)=D^{\prime }.e^{b\ell }.\;\cos\left(2\pi l\right)+{\overset{⟶}{X}}_{b}\left(t\right), \end{array}$$

where **ℓ** controls *a*_2_ parameter, *b* deﬁnes spiral shape, and (*D*′) represents the distance between search agent and target prey as deﬁned in the following equation:

(14) $$\begin{array}{c} D^{\prime }={\vec{X}}_{b}\left(t\right)-\vec{X}\left(t\right). \end{array}$$

**ℓ** is mathematically expressed in the following equation:

(15) $$\begin{array}{c} \ell \;=\left(a_{2}\;–\;1\right)*\text{rand }+\;1, \end{array}$$

where “*a*_2_” is decreasing linearly from −1 to −2 over the successive iterations *t* and expressed as the following equation:

(16) $$\begin{array}{c} a_{2}=–\;1+t*\left(\frac{\left(–1\right)}{{\text{Iter}}_{\max}}\right)\;. \end{array}$$

The exploitation phase of the WOA is implemented with equal probabilities using the following equation:

(17) $$\begin{array}{c} \overset{⟶}{P}\left(i\;+\;1\right)=\left\{\begin{array}{cc} \text{Encircling phase }\left(9\right), & p<0.5,\\ \text{Spiral phase }\left(13\right),\; & p\geq 0.5, \end{array}\right. \end{array}$$

where *pε*  (0, 1) is randomly generated number.

## 3. Proposed Methodology

*Step 1*. Input Gray Image
*Step 2*. Preprocessing
  - Apply median filter.
  - Image resizing 256 × 256 pixels.
*Step 3*. Each clustering algorithm IWOA, WOA, SSA, SCA utilize otsu's maximum between variance criteria as fitness function to compute multilevel threshold values.
*Step 4*. Image segmentation is performed by multilevel threshold values obtained by each algorithm.
*Step 5*. Predicted segmentation mask and segmentation accuracy is obtained for each clustering method based segmented image
*Step 6*. Extract DWT-PCA based texture features to train random forest machine learning algorithm
*Step 7*. Classify COVID-19/Non-COVID-19 disease by random forest algorithm

In Step 6, 2-level DWT with the Haar wavelet filter is used to extract features from the segmented image and then the PCA is applied to reduce the dimensions of features. Twelve DWT-PCA-based texture features extracted from each of the 160 IWOA, WOA, SSA, and SCA-based segmented images are fed into random forest for training, and random forest is tested with DWT-PCA-based texture features of each 40 IWOA, WOA, SSA, and SCA-based segmented images.

In Step 7, 12 DWT-PCA-based texture features are used as input for random forest to classify COVID-19/non-COVID-19 status of patients.

The flowchart of the proposed methodology is illustrated in Figure 1.

### 3.1. The Proposed Metaheuristic Algorithm (IWOA)

In this section, a variant of the WOA, the improved whale optimization algorithm (IWOA) is proposed to determine the optimal thresholds for multilevel image segmentation utilizing the maximum between-class variance criteria of the Otsu method as defined in equation (2). The flowchart of the proposed algorithm, IWOA, is illustrated in Figure 2(b). In the flowchart, E1 refers to equation (21), E2 refers to equation (9), and E3 refers to equations (18) and (19). In spiral updating position, which was discussed in Section 2.2, the WOA may trap into local optima if the best search agent or whale is far away from global solution (*X*^*∗*^).

To avoid entrapment into local optima,

(a) Search agent's position step in the WOA for |*A*| ≥ 1(exploration phase) and *p* ≥ 0.5 (spiral phase) is modified.
Updated positions of search agents for |*A* ≥ 1 under the exploration phase are mathematically modelled in the following equations:
  (18) $$\begin{array}{c} \overset{⟶}{\;D}=\left|{\overset{⟶}{P}}_{\text{rand}}-\overset{⟶}{Ps}\left(w_{\text{no}},j\right)\right|\text{.}C\text{,} \end{array}$$
  (19) $$\begin{array}{c} \overset{⟶}{P}\left(\text{t }+\;1\right)={\overset{⟶}{P}}_{\text{rand}}-\overset{⟶}{A}\overset{⟶}{D}. \end{array}$$
Here, $\overset{⟶}{Ps}\left(w\_\text{no}\right)$ represents the sorted position of whale number *w*_no at current iteration *t* and mathematically modelled in (20).
  (20) $$\begin{array}{c} w_{\text{no}}=\text{round}\left(\text{pop}-t*\left(\frac{\text{pop}-1}{T}\right)\right), \end{array}$$
Here, pop is population size of the search agent and *T* is maximum iteration.
Updated positions of search agents for *p* ≥ 0.5 is mathematically modelled in the following equation:
  (21) $$\begin{array}{c} \overset{⟶}{X}\left(t+1\right)=D^{\prime }\cdot e^{bl}.\;\cos\left(2\pi l\right)+\;\overset{⟶}{Xs}\left(t\right), \end{array}$$
where $\overset{⟶}{Xs}\left(t\right)$ represents the sorted position of whale, *b* deﬁnes the spiral shape, $\overset{⟶}{X}b\left(t\right)$ is the leader or global position of whale, and (*D*′) represents the distance between the best search agent and target prey as deﬁned in the following equation:
  (22) $$\begin{array}{c} D^{\prime }=\left|{\vec{X}}_{b}\left(t\right)-{\vec{X}}_{S}\left(t\right)\right|. \end{array}$$
Generally, **ℓ** parameter is controlled by *a*_2_ parameter, and the modification step in *a*_2_ parameter is discussed as follows.
(b) In the whale optimization algorithm (WOA), exploitation is implemented using either the encircling phase or the spiral phase. The WOA follows the best whale to converge towards global optimal solution. The WOA may trap into local optima if the best whale is far away from global solution. To avoid entrapment into local optima, randomness is introduced in the spiral phase of the WOA. Generally, **ℓ** parameter is controlled by *a*_2_ parameter as described in (15). The value of *a*_2_ parameter is dynamically selected and lies between (−1, −2); that is, the value of *a*_2_ parameter is randomly selected in the range between [−1, −2] and may obtain a random value close to −2 at starting iterations (*t*) rather than linearly decreasing (−1 to −2) over the course of iterations. *a*_2_ parameter is mathematically modelled in the following equation:
  (23) $$\begin{array}{c} a_{2}\;=-1+\left(-2+1\right)*\text{rand}\left(\right)\text{.} \end{array}$$
Now, **ℓ** parameter follows randomization in selection of its value in the spiral phase and avoids the possibility of trapping into local optima, premature convergence during the exploitation phase of the WOA.

The efficacy of the proposed algorithm is described in Section 4.2 and found that the exploration and exploitation capability of the WOA could be enhanced and chances to obtain global positions of the search agent are high over successive iterations.

The flowchart of the proposed metaheuristic clustering algorithm (IWOA) is illustrated in Figure 2(b).

## 4. Experiments and Discussion

### 4.1. Experimental Setting

The efficiency of the proposed method, IWOA, is compared with WOA, SSA, and SCA and discussed in Section 4.2. Optimal thresholds are computed by the proposed methods, IWOA, WOA, SSA, and SCA, for multilevel chest CT scan image segmentation, which is presented in Section 4.3. All algorithms are programmed in “MATLAB 2019 a” and implemented in Windows 8 64-bit computer having Intel Core i3 @ 2 GHz, 4 GB RAM. Objective function's best score, worst score, best threshold values, and segmentation measures of the proposed algorithm (IWOA) are compared with the other three algorithms, WOA [14], SSA [17], and SCA [18]. Each algorithm is tested on every image over 30 runs. For each run, whale/search agent population size and maximum iterations are set as 30 and 100, respectively, for threshold number *k* = 3. Algorithm parameters are listed in Table 1.

### 4.2. Performance of IWOA on Standard Benchmark Problems

The efficacy of the IWOA is validated on twenty-three benchmark functions; that is, unimodal (F1–F7), multimodal (F8–F13), and fixed-dimension multimodal (F14–F23), and the results are compared with other nature-inspired algorithms, namely WOA [14], SSA [17], and SCA [18].

The computation complexity of IWOA, WOA, SSA, and SCA is defined as *O* (*N* × Iter_max_) where Iter_max_ and *N* represent the maximum number of iterations and swarm population size, respectively.

In the literature, the WOA [14] has outperformed PSO, DE, FEP, and gravitational search algorithm (GSA). The SSA [17] has outperformed PSO, GSA, FPA, FA, BAT, SMS, and GA. The SCA [18] has outperformed PSO, GA, FPA, and BAT. Therefore, the computation results of PSO, DE, GSA, GA, FPA, BAT, and firefly (FA) are not included in this article.

Table 2 presents the best and worst fitness score obtained by executing each algorithm over 30 runs and 100 iterations under each run. Table 2 indicates that the IWOA and WOA both obtained similar fitness score and attained a maximum value for unimodal functions F1–F7 and multimodal F11–F13, but the IWOA achieved fast convergence and takes less number of iterations to obtain better fitness score than WOA, SSA, and SCA. The IWOA has achieved fast convergence behavior for F1–F6. SCA performed better for F7 followed by SSA, IWOA, and WOA. The IWOA obtained the best fitness score and fast convergence for F8, F9, and F10 fitness functions followed by WOA, SSA, and SCA, as shown in Figures 3–5.

Fitness functions F4, F14, F16, and F18 have similar fitness score for all algorithms over 30 runs. Overall, the IWOA achieved fast convergence and best score 11 times for F1, F2, F3, F5, F6, and F8–F13. For fitness functions F2, F3, and F13, the IWOA comes at first rank followed by the WOA at the second rank, SSA, and SCA. For fitness functions F1, F5, F6, F11, and F12, the IWOA achieved the first rank followed by the WOA (second rank), and SCA and SSA on the basis of fast convergence and best fitness score, respectively. SSA achieved fast convergence, best score, and first rank 6 times for fitness functions (F17, F19 to F23). For F19 and F20, SSA achieved first rank followed by IWOA, WOA, and SCA. For F21 to F23, SSA achieved first rank followed by SCA, IWOA, and WOA. SCA achieved the first rank twice for F7 due to the best score and fast convergence and for F18 due to fast convergence behavior.

The IWOA achieved fast convergence and best score and attains first rank for 11 fitness functions (F1–F3, F5, F6, and F8–F13) followed by the WOA as second rank. The IWOA attains the second rank 3 times for fitness functions F18, F19, and F20. Exploitation and exploration capability of all algorithms have been evaluated with unimodal (F1–F7) and multimodal (F8–F23) functions, respectively. It can be seen from Table 2 that the IWOA is a competitive and efficient optimizer for unimodal and multimodal functions and at least second in most cases.

Thus, it can be said that the proposed method, IWOA, has better exploitation and exploration capability and could avoid entrapment into local optima as compared to the considered methods. The convergence behavior of F2, F9, F6, F10, F8, and F21 is shown in Figure 3 to Figure 8 respectively, for IWOA, WOA, SSA, and SCA.

### 4.3. Benchmark Images

Performance of the proposed method (IWOA) and other methods (WOA, SSA, and SCA) utilized Otsu's maximum between variance criteria as fitness function for COVID-19 and normal chest CT scan image segmentation at threshold number *k* = 3 is evaluated on 200 randomly selected images from dataset1 [29] and dataset2 [30]. Each image has binary segmentation mask for dataset1. The image of dataset2 is resized to 256 × 256, and a binary segmentation mask is generated by simple linear iterative clustering (SLIC). Segmentation metrics from ground truths are computed.

Some sample of gray scale images (Img001.png, Img008.png, Img023.png, Img050.png, Img056.png, Img061.png, Img072.png, Img075.png, Img080.png, Img091.png) from dataset1 [29] and sample of gray images (NonCovid4.png, NonCovid31.png, NonCovid79.png, NonCovid96.png, NonCovid109.png from dataset2 [30], named SImg 1 to SImg 15, respectively, are shown in Figure 9.

### 4.4. Experimental Results and Discussion

Best fitness score (maximum fitness) and worst fitness score (minimum fitness) computed by the proposed method, IWOA, along with WOA, SSA, and SCA utilizing Otsu's maximum between variance criteria for every image at threshold number *k* = 3 are computed over 30 independent runs, and 100 iterations under each run are set for each algorithm, and the computation result of sample image is illustrated in Table 3.

Multilevel optimal threshold value is computed by each method at threshold number *k* = 3 of each image over 30 runs and optimal threshold values of sample image is illustrated in Table 4.

Quantitative metrics such as accuracy, sensitivity, specificity, precision, F_measure, *G*mean, and SSIM are computed between segmented images by each method (IWOA, WOA, SSA, and SCA), and the respective ground truth/segmentation mask under each run and segmentation metrics for each image is computed by each method. Segmentation metrics for 15 sample images computed by each method is listed in Tables 5–8 as an average of 30 runs and further average segmentation metrics of 15 images are computed.

It is clear from Tables 5–8 that the average segmentation metrics computed for 15 IWOA-based sample segmented images are better than those of the segmented images computed based on the other methods. Segmentation metrics such as accuracy, sensitivity, specificity, precision, *F*_measure, and *G*mean are computed between binary segmentation image mask (predicted binary mask) and binary segmentation mask (ground truth) of the corresponding image from the dataset. SSIM is computed between gray-level segmentation image mask (predicted binary mask) and gray-level segmentation mask (ground truth) of the corresponding image from the dataset. Average segmentation metrics computed for 15 IWOA-, WOA-, SSA-, SCA-based segmentation images are compared and listed in Table 9 and shown in Figure 10. It is clear from Table 9 that the IWOA has achieved 1st rank in segmentation measures followed by SSA (2nd rank), WOA, (3rd rank), and SCA (4th rank).

Discrete wavelet transform (DWT) and principal component analysis (PCA) are applied on each of the 200 IWOA-, WOA-, SSA-, and SCA-based segmented images over 30 runs to extract the first-order and second-order texture features. Two-level DWT with the Haar wavelet filter is used to extract features from the segmented image, and then, PCA is applied to reduce the dimensions of features. PCA selects the important ordered feature set. Twelve DWT-PCA-based texture features extracted from each 15 IWOA-based segmented images (SegImg1 to SegImg15) are listed in Table 10 as an average of 30 runs, and further average texture features are computed. Second-order texture features [31] such as correlation, contrast, homogeneity, and energy are computed by the GLCM pattern. Twelve DWT-PCA-based texture features extracted from each of the 160 IWOA-, WOA-, SSA-, and SCA-based segmented images are fed into random forest [32] for training. Random forest is tested with DWT-PCA-based texture features of each of 40 IWOA-, WOA-, SSA-, and SCA-based segmented images. Twelve DWT-PCA-based texture features are used as input for random forest to classify COVID-19/Non-COVID-19 status of patients. Random forest has achieved promising 97.49% classification accuracy for DWT-PCA-based texture features of IWOA-based segmented image.

The visual quality of the predicted segmentation mask, RGB-labelled segmented image, and segmented image for the best threshold value computed by the proposed method (IWOA) along with WOA, SSA, and SCA is shown in Figure 11. The IWOA method achieves better segmentation accuracy and visual quality of predicted segmentation mask and segmented image than other methods.

Table 11 indicates that the predicted segmentation mask generated by the IWOA method for SImg2, SImg3, SImg13, and SImg15 has achieved better segmentation accuracy compared to the predicted segmentation mask generated by other methods.

From Table 12, it is inferred that the random forest algorithm has achieved promising 97.49% classification accuracy for DWT-PCA-based texture features, which are extracted from IWOA-based segmented images. When the texture features are extracted from SSA-based segmented images, the random forest achieved 94.12% accuracy, which further decreased by 1% if the texture features are extracted from WOA-based segmented images. Random forest has given the least accuracy 90% for DWT-PCA-based texture features, which are extracted from SCA-based segmented images.

## 5. Conclusion

Diagnosing COVID-19 disease through an RT-PCR test is a time-consuming process, and sometimes, the RT-PCR test has a false-negative result, which can cause a threat to the person's life due to delay in starting the specified treatment. At this moment, there is an urgent need to develop an automatic COVID-19 detection tool that can detect the COVID-19 disease from chest CT scan images within a shorter span of time. In this article, a variant of the existing whale optimization algorithm named improved whale optimization algorithm (IWOA) is introduced to compute optimal threshold values. The efficiency of the IWOA is tested using 23 benchmark optimization functions, and it was proven that the IWOA achieved better convergence behavior, and improved the exploitation and exploration ability of WOA and bypass local optima. The proposed method (IWOA) and WOA, SSA, and SCA as clustering methods utilize Otsu's maximum between-class variance criteria to compute the optimal threshold. Automated segmentation is performed with optimal threshold values (*k* = 3). The IWOA method has achieved a better fitness score, segmentation accuracy, visual quality of predicted segmentation mask, and segmented image than other methods. The IWOA-based segmentation method grips the 1st rank to evaluate segmentation metrics. Two-level DWT with the Haar wavelet filter is used to extract the features from the segmented image, and then, PCA is applied to reduce dimensions of features. Twelve DWT-PCA texture features extracted from the segmented image are utilized as input to the random forest machine-learning algorithm for the classification of COVID-19/Non-COVID disease. The random forest algorithm has reported a promising classification accuracy of 97.49% for DWT-PCA-based texture features, which are extracted from IWOA-based segmented images. In the future, DWT-PCA-based texture features extracted from the proposed method will be fed as input to various machine-learning and pretrained deep learning models to detect tumour from brain MRI images and classification metrics comparison will be carried out.

## Figures and Tables

**Figure 1:** Flowchart of the proposed methodology.

**Figure 2:** (a) Variation in *a*_2_ parameter. (b) Flowchart of the proposed metaheuristic clustering algorithm (IWOA).

**Figure 3:** Convergence behavior of fitness function F2.

**Figure 4:** Convergence behavior of fitness function F9.

**Figure 5:** Convergence behavior of fitness function F6.

**Figure 6:** Convergence behavior of fitness function F10.

**Figure 7:** Convergence behavior of fitness function F8.

**Figure 8:** Convergence behavior of fitness function F21.

**Figure 9:** Samples of gray scale images from SImg1 to SImg15.

**Figure 10:** Comparison of average segmentation metrics of IWOA, WOA, SSA, and SCA.

**Figure 11:** Predicted segmentation mask, labelled segmented image, and segmented image for the best threshold value computed by the proposed method (IWOA) and WOA, SSA, and SCA.

**Algorithm 1:** Whale optimization algorithm (WOA) [14].

**Table 1:** Parameters of each algorithm.

Algorithm/method	Parameters	Value
Improved whale optimization algorithm (IWOA)	*a*_1_	2 to 0
	*a*_2_	[−1, −2]
	*b*	1
	**ℓ**	[−1, 1]
Whale optimization algorithm (WOA)	*a*_1_	2 to 0
	*a*_2_	−1 to −2
	*B*	1
	**ℓ**	[−1, 1]
Salp swarm algorithm (SSA)	*c*_1_	2 to 0
Sine cosine algorithm (SCA)	*A*	2
	*r*_1_, *r*_2_, *r*_3_, *r*_4_	[0, 1]
Dim (Threshold number)	*k*	3
Upper bound Xmax	UB	255
Lower bound Xmin	LB	0

**Table 2:** The best and worst fitness values over 30 runs.

	WOA		IWOA		SSA		SCA	
	Best	Worst	Best	Worst	Best	Worst	Best	Worst
F1	**3.0E** **+** **05**	**3.0E** **+** **05**	**3.0E** **+** **05**	**3.0E** **+** **05**	2.71*E* + 05	2.48*E* + 05	2.75*E* + 05	2.52*E* + 05
F2	**1.0E** **+** **30**	**1.0E** **+** **30**	**1.0E** **+** **30**	**1.0E** **+** **30**	3.41*E* + 29	1.09*E* + 29	2.01*E* + 28	0.703*E* + 28
F3	**9.45E** **+** **07**	**9.45E** **+** **07**	**9.45E** **+** **07**	**9.45E** **+** **07**	7.64*E* + 07	6.04*E* + 07	4.73*E* + 07	3.20*E* + 07
F4	100	100	100	100	100	100	100	100
F5	**2.50E** **+** **09**	**2.50E** **+** **09**	**2.50E** **+** **09**	**2.50E** **+** **09**	1.92*E* + 09	1.80*E* + 09	2.07*E* + 09	1.89*E* + 09
F6	**3.03E** **+** **05**	2.97*E* + 05	**3.03E** **+** **05**	**3.03E** **+** **05**	2.60*E* + 05	2.48*E* + 05	2.62*E* + 05	2.50*E* + 05
F7	1249	1249	1249	1249	2332	1605	**2543**	**1660**
F8	8041	7701	**8778**	**8600**	7156	5738	4334	2898
F9	1199	1072	**1204**	**1193**	972	880	848	832
F10	22.09	21.90	**22.31**	**21.98**	21.92	21.83	21.57	21.47
F11	**2701**	**2701**	**2701**	**2701**	2331	2163	2420	2266
F12	**7.68E** **+** **09**	**7.68E** **+** **09**	**7.68E** **+** **09**	**7.68E** **+** **09**	6.06*E* + 09	5.55*E* + 09	6.67*E* + 09	5.85*E* + 09
F13	1.23*E* + 10	1.23*E* + 10	1.23*E* + 10	1.23*E* + 10	1.09*E* + 10	0.98*E* + 10	1.01*E* + 10	0.94*E* + 10
F14	499.99	499.99	499.99	499.99	499.99	499.99	499.99	499.99
F15	Inf	Inf	Inf	Inf	Inf	Inf	Inf	Inf
F16	6400	6400	6400	6400	6400	6400	6400	6400
F17	308	308	308	308	**505**	308	308	308
F18	1.01*e* + 06	1.01*e* + 06	1.01*e* + 06	1.01*e* + 06	1.01*e* + 06	1.01*e* + 06	**1.01e** **+** **06**	**1.01e** **+** **06**
F19	−0.068	−0.068	−0.068	−0.068	−**0.37E** − **04**	−**0.37E** − **04**	−0.068	−0.068
F20	−0.0051	−0.0051	−0.0051	−0.0051	−**0.27E** − **07**	−**0.27E** − **07**	−0.0051	−0.0051
F21	−0.0412	−0.0412	−0.0412	−0.0412	−**0.0377**	−**0.0377**	−0.0377	−0.0377
F22	−0.0504	−0.0504	−0.0504	−0.0504	−0.0504	−0.0504	−0.0504	−0.0504
F23	−0.0784	−0.0784	−0.0784	−0.0784	−0.0784	−0.0784	−0.0784	−0.0784

Bold entries represent the best value.

**Table 3:** Best and worst fitness scores of various algorithms.

Images	Best fitness values				Worst fitness values			
	WOA	IWOA	SSA	SCA	WOA	IWOA	SSA	SCA
SImg 1	2723	2725	2723	2721	2723	2724	2721	2712
SImg 2	3462	3462	3462	3459	3460	3462	3462	3454
SImg 3	3330	3332	3332	3328	3329	3334	3332	3325
SImg 4	4165	4165	4165	4162	4163	4165	4165	4158
SImg 5	600	605	603	596	600	602	601	562
SImg 6	2772	2778	2774	2772	2770	2773	2772	2770
SImg 7	1568	1575	1572	1568	1566	1573	1573	1566
SImg 8	2234	2238	2236	2233	2229	2234	2232	2229
SImg 9	1378	1384	1384	1377	1374	1382	1382	1374
SImg 10	1186	1190	1189	1185	1181	1188	1188	1180
SImg 11	1945	1948	1946	1945	1943	1947	1945	1943
SImg 12	2372	2384	2380	2372	2370	2382	2376	2369
SImg 13	1682	1689	1688	1681	1679	1684	1684	1678
SImg 14	2165	2170	2170	2163	2163	2168	2168	2163
SImg 15	1744	1749	1747	1743	1741	1746	1745	1741

**Table 4:** Best threshold values of various segmentation methods.

Image	IWOA	WOA	SSA	SCA
SImg 1	35,50,66	25,36,227	75,192,242	70,188,234
SImg 2	124,139,198	8,27,36	22,68,254	45,133,194
SImg 3	55,143,218	31,52,121	57,94,254	65,143,213
SImg 4	20,133,238	102,109,133	18,50,254	39,156,211
SImg 5	31,235,244	40,114,164	31,58,174	45,174,198
SImg 6	18,35,179	137,162,253	65,200,234	56,124,189
SImg 7	60,205,249	85,152,249	67,110,254	70,137,221
SImg 8	81,171,249	135,184,208	61,185,242	58,134,197
SImg 9	30,125,224	17,170,181	12,34,143	60,124,168
SImg 10	3,21,92	8,33,204	4,27,154	10,65,188
SImg 11	122,224,246	101,178,186	10,183,234	39,126,254
SImg 12	143,151,214	118,138,211	44,113,194	10,138,214
SImg 13	122,143,252	141,216,249	4,81,201	25,127,214
SImg 14	116,135,196	104,200,216	4,78,157	42,59,187
SImg 15	148,168,234	172,182,231	26,153,179	47,145,254

**Table 5:** Quantitative metrics by the IWOA.

Image	Accuracy	Sensitivity	Specificity	Precision	*F*_measure	*G*mean	SSIM
SImg 1	0.9804	0.8934	0.9956	0.9728	0.9314	0.9431	0.9509
SImg 2	0.9666	0.9032	0.9913	0.9758	0.938	0.9462	0.8701
SImg 3	0.9732	0.9282	1	1	0.9627	0.9634	0.9111
SImg 4	0.9865	0.6588	0.9959	0.8246	0.7324	0.81	0.9344
SImg 5	0.9399	0.786	0.9919	0.9705	0.8685	0.883	0.8037
SImg 6	0.9114	0.7672	0.9773	0.9392	0.8445	0.8659	0.7109
SImg 7	0.9508	0.6875	0.985	0.8632	0.7653	0.8231	0.8028
SImg 8	0.9924	0.7259	0.9964	0.7597	0.7424	0.8505	0.9662
SImg 9	0.94	0.7853	0.9924	0.9724	0.8688	0.8828	0.8402
SImg 10	0.9642	0.6448	0.9921	0.8772	0.7432	0.7998	0.8303
SImg 11	0.9954	0.9875	1	1	0.9937	0.9937	0.8003
SImg 12	0.9906	1	0.9832	0.9794	0.9896	0.9916	0.8920
SImg 13	0.9926	0.9886	1	1	0.9943	0.9943	0.9227
SImg 14	0.9742	0.9528	1	1	0.9758	0.9761	0.9517
SImg 15	0.9840	1	0.9673	0.9699	0.9847	0.9835	0.8504
**Avg.**	**0.9695**	**0.8472**	**0.9912**	**0.9403**	**0.8890**	**0.9138**	**0.8691**

Bold entries represent the average value of 15 images.

**Table 6:** Quantitative metrics by WOA.

Image	Accuracy	Sensitivity	Specificity	Precision	*F*_measure	*G*mean	SSIM
SImg 1	0.9324	0.9006	0.9355	0.5687	0.6971	0.9178	0.8286
SImg 2	0.9149	0.9076	0.9169	0.7481	0.8201	0.9122	0.6945
SImg 3	0.8815	0.4835	0.9998	0.8627	0.6197	0.6953	0.9568
SImg 4	0.9862	0.6705	0.9926	0.6780	0.6742	0.8158	0.9120
SImg 5	0.8866	0.6069	0.9012	0.5425	0.5729	0.7395	0.7699
SImg 6	0.7578	0.7017	0.6026	0.5663	0.6268	0.6503	0.6104
SImg 7	0.9046	0.4396	0.9141	0.7950	0.5661	0.6339	0.7440
SImg 8	0.9693	0.8207	0.9903	0.3343	0.4751	0.9015	0.9582
SImg 9	0.9275	0.9231	0.9051	0.5976	0.7255	0.9140	0.7470
SImg 10	0.9628	0.7893	0.9696	0.5044	0.6154	0.8748	0.8359
SImg 11	0.9705	0.9246	1	1	0.9608	0.9615	0.7500
SImg 12	0.9905	0.9796	1	1	0.9897	0.9897	0.7900
SImg 13	0.9894	1	0.9715	0.9834	0.9916	0.9856	0.9037
SImg 14	0.9172	0.8627	1	1	0.9263	0.9288	0.8163
SImg 15	0.9720	1	0.9439	0.9471	0.9728	0.9715	0.6242
**Avg,**	**0.9309**	**0.8007**	**0.9362**	**0.7419**	**0.7489**	**0.8595**	**0.7961**

Bold entries represent the average value of 15 images.

**Table 7:** Quantitative metrics by SSA.

Images	Accuracy	Sensitivity	Specificity	Precision	F_measure	*G*mean	SSIM
SImg 1	0.8692	0.8839	0.8722	0.7797	0.8285	0.8780	0.8077
SImg 2	0.9635	0.9062	0.9852	0.9587	0.9317	0.9449	0.8267
SImg 3	0.9862	0.9875	0.7770	0.5299	0.6897	0.8759	0.9560
SImg 4	0.9546	0.3219	0.9982	0.9270	0.4779	0.5669	0.9103
SImg 5	0.9106	0.5872	0.9904	0.9381	0.7223	0.7626	0.7976
SImg 6	0.8097	0.7875	0.8670	0.4299	0.5562	0.8263	0.5781
SImg 7	0.8590	0.6553	0.9971	0.9760	0.7841	0.8083	0.8133
SImg 8	0.9893	0.8207	0.9903	0.3343	0.4751	0.9015	0.9581
SImg 9	0.9400	0.9702	0.9323	0.7866	0.8688	0.9511	0.7280
SImg 10	0.9185	0.4144	0.9950	0.9277	0.5729	0.6422	0.8300
SImg 11	0.9715	1	0.9573	0.9213	0.959	0.9781	0.8976
SImg 12	0.9670	1	0.9431	0.9271	0.9621	0.9711	0.7480
SImg 13	0.9339	0.8967	1	1	0.9455	0.9469	0.6987
SImg 14	0.9742	1	0.9490	0.9504	0.9746	0.9741	0.8765
SImg 15	0.9809	1	0.9611	0.9640	0.9816	0.9803	0.8996
**Avg.**	**0.9352**	**0.8154**	**0.9477**	**0.8234**	**0.7820**	**0.8672**	**0.8217**

Bold entries represent the average value of 15 images.

**Table 8:** Quantitative metrics by SCA.

Images	Accuracy	Sensitivity	Specificity	Precision	*F*_measure	*G*mean	SSIM
SImg 1	0.8710	0.7116	0.8740	0.6327	0.6698	0.7886	0.80772
SImg 2	0.7510	0.8423	0.7496	0.9058	0.8729	0.7946	0.6578
SImg 3	0.9721	0.6271	0.7865	0.8123	0.7078	0.7023	0.9515
SImg 4	0.9532	0.3156	0.9983	0.9331	0.4712	0.5613	0.9097
SImg 5	0.9245	0.6349	0.9879	0.9199	0.7513	0.7919	0.8000
SImg 6	0.7331	0.7479	0.7416	0.5784	0.6523	0.7448	0.5862
SImg 7	0.9446	0.5505	0.9875	0.4396	0.4888	0.7373	0.8133
SImg 8	0.9493	0.8207	0.9903	0.3343	0.4751	0.9015	0.9582
SImg 9	0.7959	0.6470	0.7962	0.5574	0.5989	0.7177	0.7279
SImg 10	0.9628	0.7893	0.9696	0.5044	0.6154	0.8748	0.8359
SImg 11	0.9984	0.9957	1	1	0.9978	0.9978	0.9893
SImg 12	0.9935	1	0.9883	0.9857	0.9927	0.9941	0.6969
SImg 13	0.7653	1	0.6055	0.6332	0.7754	0.7781	0.6184
SImg 14	0.9426	0.8897	1	1	0.9416	0.9432	0.7043
SImg 15	0.9671	0.9415	1	1	0.9698	0.9703	0.7456
**Avg.**	**0.9016**	**0.7676**	**0.8983**	**0.7491**	**0.7320**	**0.8199**	**0.7868**

Bold entries represent the average value of 15 images.

**Table 9:** Comparison of average segmentation metrics of IWOA, WOA, SSA, and SCA.

Segmentation measures	Methods			
	IWOA	WOA	SSA	SCA
Accuracy	**0.9695**	0.9309	0.9352	0.9016
Specificity	**0.9912**	0.9362	0.9477	0.8983
Precision	**0.9403**	0.7419	0.8234	0.7491
Sensitivity	**0.8472**	0.8007	0.8154	0.7676
*F*_measure	**0.8890**	0.7489	0.7820	0.7320
*G*mean	**0.9138**	0.8595	0.8672	0.8199
SSIM	**0.8691**	0.7961	0.8217	0.7868

Bold entries represent the best value.

**Table 10:** DWT-PCA-based texture features of IWOA-based segmented image.

Features	Images							
	SegImg 1	SegImg 2	SegImg 3	SegImg 4	SegImg 5	SegImg 6	SegImg 7	SegImg 8
Contrast	0.1197	0.1020	0.1387	0.1217	0.1202	0.0932	0.1172	0.1503
Correlation	0.9778	0.8647	0.9669	0.9660	0.6612	0.9736	0.8898	0.8059
Homogeneity	0.9733	0.9739	0.9740	0.9733	0.9746	0.9702	0.9716	0.9774
Mean	0.00151	0.00087	0.00252	0.00210	0.00202	0.00115	0.00178	0.0018
Std. deviation	0.06017	0.06018	0.06014	0.06015	0.06016	0.06018	0.06016	0.06016
Variance	0.003621	0.003622	0.003623	0.00362	0.00362	0.003619	0.003621	0.003624
Entropy	2.140	2.6620	1.5241	1.8340	2.3087	2.7367	2.3822	1.0632
Energy	0.9012	0.9018	0.9068	0.9001	0.9060	0.8855	0.8946	0.9204
Smoothness	0.9659	0.9424	0.9792	0.9752	0.9743	0.9557	0.9710	0.9714
Kurtosis	26.65	23.53	31.46	27.60	31.62	17.14	29.79	43.02
Skewness	1.7083	1.3639	2.2488	1.7548	2.1902	0.9658	1.8319	2.5913
IDM	1.3841	1.7791	−0.5052	1.425	2.790	−0.3163	1.2450	0.6260

Features	SegImg 9	SegImg 10	SegImg 11	SegImg 12	SegImg 13	SegImg 14	SegImg 15	Avg.

Contrast	0.1145	0.1112	0.0779	0.0827	0.0883	0.0825	0.0860	0.107073
Correlation	0.9853	0.9534	0.9543	0.9500	0.9186	0.9355	0.9454	0.91656
Homogeneity	0.9740	0.9726	0.9710	0.9710	0.9719	0.9711	0.9702	0.972673
Mean	0.00092	0.00151	0.00071	0.00122	0.00093	0.00137	0.00152	0.001462
Std. deviation	0.06018	0.06017	0.06019	0.06018	0.06018	0.06017	0.06017	0.060169
Variance	0.003621	0.003622	0.003618	0.003618	0.003618	0.003614	0.003619	0.00362
Entropy	2.3972	2.1250	3.1821	3.0411	2.9107	3.2324	3.1900	2.448627
Energy	0.90291	0.89888	0.88843	0.88816	0.89214	0.89083	0.88684	0.897639
Smoothness	0.9454	0.9660	0.9306	0.9582	0.9459	0.9625	0.9662	0.96066
Kurtosis	24.34	24.79	7.80	10.36	15.01	9.05	9.58	22.116
Skewness	1.5156	1.5021	0.3749	0.5657	0.7329	0.6256	0.6490	1.37472
IDM	1.2370	1.7377	−0.0899	0.6499	0.7130	1.2152	−0.6299	0.884047

**Table 11:** Segmentation accuracy of predicted segmentation mask.

Images	IWOA	WOA	SSA	SCA
SImg2	**97.98**	93.23	96.49	74.59
SImg3	**98.34**	95.39	96.68	76.83
SImg13	**98.56**	96.78	95.54	90.12
SImg15	**97.59**	96.63	96.89	92.47

Bold entries represent best value.

**Table 12:** Comparative analysis of classification metric.

Method/References	Description	Classification model/tool	Metric
IWOA	DWT-PCA texture features from the IWOA-based segmented image	Random forest	**Accuracy: 97.49%**
WOA	DWT-PCA texture features from the WOA-based segmented image	Random forest	Accuracy: 93.26%
SSA	DWT-PCA texture features from the SSA-based segmented image	Random forest	Accuracy: 94.12%
SCA	DWT-PCA texture features from SCA-based segmented image	Random forest	Accuracy: 90%
Reference [6]	Fine-tuned DL architectures to detect COVID-19 from chest X-ray images	DenseNet121	Accuracy: 97%
		Xception	Accuracy: 96%
		MobileNetv2	Accuracy: 95%
		ResNet50v2	Accuracy: 94%
		VGG19	Accuracy: 92%
		Inceptionv3	Accuracy: 90%
Reference [8]	COVID-19 lung CT image segmentation to assess the diagnosis of COVID-19 patients	SegNet	Accuracy: 95%
		U-NET	Accuracy: 91%
Reference [9]	Identification of COVID-19 images from chest X-rays using DL	Cognex's Vision Pro DL software	*F*-Score: 94%

Bold entries represent the best value.

## Data Availability

The simulation experiment method used to compute the findings is available from the corresponding author upon request.

## Abbreviations

COVID-19: Coronavirus disease-19
RT-PCR: Reverse-transcription polymerase chain reaction
DL: Deep learning,
PCA: Principal component analysis
IDM: Inverse difference moment
DWT: Discrete wavelet transform.
